The article "Information Dissemination Model in Rural Live Broadcasting under Blockchain in the Era of Artificial Intelligence" was retracted in 2023. Reasons: unreliable results or conclusions; concerns about the data; concerns about the peer review; concerns about the citations.

# Information Dissemination Model in Rural Live Broadcasting under Blockchain in the Era of Artificial Intelligence

**DOI:** 10.1155/2022/4590578

**Published:** 2022-07-11

**Authors:** Jie Liu, Yahui Yu, Peng Ji, Danni Liu

**Affiliations:** ^1^Shanxi Normal University, Taiyuan, China; ^2^Shanxi Vocational College of Art, Taiyuan 030000, China; ^3^Communication University of Shanxi, Taiyuan 030000, China; ^4^Shanxi College of Application Science and Technology, Taiyuan 030000, China

## Abstract

This work aims to improve the information dissemination atmosphere of rural live broadcasting and ensure its long-term development. First, it studies and analyzes the current situation and characteristics of rural live broadcasting. Then, it discusses the blockchain (BC) technology and information dissemination mode in the era of artificial intelligence (AI). Finally, the characteristics of BC technology (BT) and the information dissemination model are discussed. A BT-optimized susceptible exposed infected recovered (SEIR) information dissemination model is proposed. The results show that the BT-optimized SEIR model has no effect on the traditional information transmission characteristics and can ensure the conventional transmission of all information. Additionally, BT can effectively improve the overall transmission efficiency of the SEIR model for false information and accurate information and effectively shorten the duration. Specifically, the BT-optimized SEIR model's maximum false information transmission proportion is reduced by about 13%. The duration is reduced by 15 days over the traditional model. By comparison, in positive information dissemination, the maximum transmission proportion of the proposed BT-optimized SEIR model is about 19% higher than the traditional model. The duration is about 30 days longer. The research provides technical support for controlling and improving the current situation and atmosphere of rural live broadcasting information dissemination.

## 1. Introduction

Artificial intelligence (AI) technology has become the mainstream science and technology in today's society. For example, many intelligent network technologies are widely used in human life and daily activities. AI studies and develops theories, methods, technologies, and application systems to simulate, regenerate, and expand human intelligence. AI aims to empower machines to listen (speech recognition (SR) and machine translation (MT)) and see (image recognition (IR) and character recognition (CR)). It also teaches computers to speak (speech synthesis and man-machine dialogue) and think (man-machine game and theorem proving). Ultimately, machines can learn (machine learning (ML) and knowledge representation (KR)) and act (robots and autonomous driving (AD)). In particular, blockchain (BC) technology excels among many network technologies. It has many advantages, such as decentralization, distrust, security, reliability, and traceability. Thus, BC technology (BT) has been popularized in the social environment [1]. Meanwhile, rural live streaming is becoming one of the main factors affecting rural development. Nevertheless, some misconducts need to be improved, and moral and legal standards must be formulated. In order to do so, network technological reformation provides new enlightenment for rural live streaming sectors [2]. Although the current implementation of state-of-the-art technologies in rural development is not perfect, many studies have provided technical support.

The article "Information Dissemination Model in Rural Live Broadcasting under Blockchain in the Era of Artificial Intelligence" was retracted in 2023. Reasons: unreliable results or conclusions; concerns about the data; concerns about the peer review; concerns about the citations.

Wang and Su (2020) [3] pointed out that BT was a distributed database technology. BC was characterized by decentralization, transparency, fairness, and openness and was consistent with the Internet of Energy (IoE) concept. Thus, BC saw ever-broader applications. Hakak et al. [4] believed that BT was a distributed data recording scheme applicable to all transactions or electronic behaviors. Because of accurate information identification, BT has aroused the attention and discussion of the public from all walks of life. Sedlmeir et al. [5] said that BC was an organization that managed and maintained multiparty cooperation. Each party should establish an independent database to carry business data. The differences between multiparty databases often led to manual review and disputes. In this case, BT could solve the trust problem between multiple parties. BT could establish a reliable, tamper-proof, traceable, and multiparty distributed database among unknown parties as a decentralized system. BT could realize a point-to-point (P2P) information transmission without the coordination of third-party intermediaries. Park and Lin [6] mentioned that the development of network technology and the fusion of virtual and real economies have helped some rural areas eliminate poverty. “Selling goods through live streaming” was a critical means of getting rid of poverty and getting rich in rural areas after improving farmers' new media literacy. Whon and Freeman [7] argued that the increasing network transmission speed and audiences' demand for information timeliness, sense of the scene, and other perspectives gave birth to live streaming. Live streaming has been widely used in other live programs since it first set foot in sports events. The traditional way of relying solely on live television (TV) to obtain information changed quietly. Wongkitrungrueng and Asarut [8] reasoned that with the development of the Internet, live streaming platforms have become diversified, including computers and mobile phones. The explosive development of China's live streaming business has attracted many investments and become the fastest-growing industry. Live streaming platforms and network anchors have sprung up because information could only be released to the live streaming platform through video using simple devices. Broadcast content was designed for users, viewers, communicators, producers, and judges. Users with the same hobbies or attitudes would spontaneously form a highly participatory and interactive community with the anchor. The anchor met users' needs in exchange for interaction and rewards, so users' preferences affected the live content. In summary, although the above literature points out the defects of the current live streaming environment and explains the underlying causes, it does not put forward specific solutions. Therefore, more research is needed to comprehensively improve the current live streaming environment.

The article "Information Dissemination Model in Rural Live Broadcasting under Blockchain in the Era of Artificial Intelligence" was retracted in 2023. Reasons: unreliable results or conclusions; concerns about the data; concerns about the peer review; concerns about the citations.

Actually, nonprofessionals can also set up live streaming because of relatively low requirements on skills. This kind of live streaming provides an easy-communicative environment and receives a large variety of public with fair distribution. However, the absence of industry norms and supervision means that some problems are inevitable, causing excessive entertainment, consumption, and vulgar content. Therefore, it is necessary to improve the conditions for disseminating information. Kudchadkar and Coroll [9] claimed that new Internet applications based on social network services were developing rapidly. Social networks have become essential for people to spread information and communicate. Unlike the traditional information dissemination model, the social network had a fast dissemination speed. It could control its dissemination process, but the formation and evolution of public opinions were complex and uncertain. Thus, traditional theories and overly simplified models challenged the understanding of the evolution of public opinion in information dissemination and social networks.

According to the above literature review, this work first analyzes the current situation and characteristics of rural live broadcasting to provide a theoretical basis for the subsequent research. Then, BT and information dissemination are discussed, which provides a technical basis for the research. Finally, an information dissemination optimization model for rural live broadcasting based on BT is proposed, and the model is comprehensively evaluated. The innovation of this work is to combine network information dissemination technology with BT to provide a better and safer technical means and environment for rural live broadcasting. The research results provide technical support for optimizing information dissemination based on rural live broadcasting and help improve society's overall live broadcasting atmosphere.

The article "Information Dissemination Model in Rural Live Broadcasting under Blockchain in the Era of Artificial Intelligence" was retracted in 2023. Reasons: unreliable results or conclusions; concerns about the data; concerns about the peer review; concerns about the citations.

## 2. Theories and Methods

### 2.1. Rural Information Dissemination

The development of the Internet and various network technologies brings countless benefits to human society and also poses many threats. Social networks provide a broad communication platform for humankind and change people's communication methods. Traditional face-to-face communication is changed into the current information exchange, video exchange, and live communication with the help of social networks. However, some criminals take advantage of the communication mode to earn ill-gotten money [10]. In view of this, live broadcasting is also becoming the most harmful online social mode to the public. The reason is that people can communicate online without their real names or anonymously. Alternatively, they can beautify themselves through different costumes and plug-ins through social software. These behaviors make the online social platform difficult to distinguish the true information from the false in the communication process. Anonymity or a false identity makes many people unscrupulous, spread information indiscriminately, disturb social networks' order, and even engage in illegal and criminal activities [11].

Based on social networks, the information in both cities and rural areas is spread rapidly through live broadcasting. However, many people in rural areas do not receive much education. They have little knowledge of social networks, resulting in disclosing important personal information and being cheated by some false information. Live broadcasting is originally a sociable way to improve the communication efficiency of culture, knowledge, and positive energy. However, the current live broadcasting network has caused significant damage to audiences' interests due to inadequate supervision in information dissemination and transactions [12]. Rewarding is the most direct way for the anchor to make money, so many anchors gain rewordings by spreading inappropriate information or artificial commodities. The live broadcast software only provides the platform for the audience and the anchor. It draws a commission from the live broadcast revenue of the anchor, but it does not bear the risks brought by the live broadcast. Moreover, some supervision measures are not implemented after the audience rewards, so the audience's rights and interests cannot be protected or guaranteed [13].  Figure 1 shows the operating principle of the live broadcast platform.

The article "Information Dissemination Model in Rural Live Broadcasting under Blockchain in the Era of Artificial Intelligence" was retracted in 2023. Reasons: unreliable results or conclusions; concerns about the data; concerns about the peer review; concerns about the citations.

Figure 1 shows that the anchor and the audience are direct participants in live broadcasting. The audience rewards the anchor. Society begins to spread information about characteristic rural products for rural people, especially when the sale of characteristic agricultural products is suspended under the epidemic's impact. Therefore, live selling successfully meets the urgent needs of peasants and helps them obtain the anticipated benefits [14]. Peasants, public welfare anchors, and others can all sell products on live broadcasting platforms [15].  Figure 2 shows the main channels, through which agricultural products are sold in live broadcasting.

Figure 2 shows that buying agricultural products on the live broadcasting platform is one of the main ways to help peasants get rid of poverty. Therefore, a rural live broadcasting style is formed in rural areas to market agricultural products, promote the brand, and publicize agricultural products' planting and breeding process [16]. Through TikTok marketing, agricultural products are sold through the function of “friends” of WeChat, microblog, jitter, and other software platforms. Netizens pick up the commodities in the live broadcast through the anchors' introduction and then place an order, becoming a common way to sell goods. Brand promotion means that agricultural products are advertised on some APPs. The sales of their offline and online agricultural products are growing fast. The government generally supports the traditional brand promotion of agricultural products undertaken by enterprises and peasants on television, newspapers, and radio. This method has a high cost but a low effect, so the annual income of peasants is also short [17]. Now, the promotion activities of agricultural product brands are conducted via network channels, improving the promotion efficiency and reducing the cost. Therefore, the promotion on network platforms is also one of the main ways to create agricultural product brands [18]. Publicizing the planting and breeding process of agricultural products through live broadcasting is another way for peasants to sell their agricultural products. Thus, peasants can showcase the agricultural production details to alleviate netizens' food safety concerns. Doing so improves the peasant's popularity and favor and achieves the ultimate goal of online live selling [19]. Moreover, peasants with professional knowledge and planting experience can spread their planting and breeding processes to others through live broadcasting. This meets the market's needs and successfully increases peasants' income [20].  Figure 3 shows the current mode of rural live broadcasting and its primary functions.

The article "Information Dissemination Model in Rural Live Broadcasting under Blockchain in the Era of Artificial Intelligence" was retracted in 2023. Reasons: unreliable results or conclusions; concerns about the data; concerns about the peer review; concerns about the citations.

Figure 3 shows that rural live broadcasting is related to the sales and publicity of agricultural products and consumers' rights and interests. In view of this, the live broadcasting platform should ensure the authenticity and effectiveness of public information and protect consumers. Therefore, an information transmission model is needed in rural live broadcasting. It has great significance to the development of rural areas [21].

## 3. Blockchain Technology

BT originates from bitcoins, a digital currency. It is the process of packaging data in chronological order through BC, connecting them according to the packaged blocks. Then, it forms a BC for data transmission and storage, achieving data security through passwords and preventing data tampering and embezzlement [22]. It has high efficiency in information transmission because it comprises countless blocks with block headers, data blocks, and block bodies. The block header includes hash values, time tags, random digital tags, and other information [23]. The data block stores the data to be transmitted. The block body contains the data to be transmitted [24].  Figure 4 shows the structure of a BC.

Figure 4 shows that data transmission through BCs can ensure data security and store the data through the time tag, which increases data utilization and comprehensively improves its efficiency. BCs have several characteristics: decentralization, distrust, nontamperability, and traceability [25]. The information transmission mode of the BC network is point to point. The information transmission nodes are separated from each other. They do not need any intermediary structure, ensuring the fairness and security of information transmission. In addition, the information transmission process is transparent throughout the network and has stored information in the BC, ensuring its traceability [26].

### 3.1. Broadcast Information Dissemination Model

The information dissemination model includes an influence model and an infectious disease model based on the game theory. The infectious disease model classifies the population according to their infection states, namely, vulnerability to infection, immunity, and infection [27]. Based on these states, the information dissemination model can be divided into the susceptible infected (SI) model, sustainable infected sustainable (SIS) model, sustainable infected recovered (SIR) model, and sustainable infected recovered sustainable (SIRS) model. The SI model includes the easily infected state and the infected state. In this model, the infected person spreads the information to the easily infected person when they contact [28]. The calculation equations of the SI model are as follows:

(1) $$\begin{array}{c} \frac{dS\left(t\right)}{dt}=-\lambda S\left(t\right)I\left(t\right), \end{array}$$

(2) $$\begin{array}{c} \frac{dI\left(t\right)}{dt}=\lambda S\left(t\right)I\left(t\right). \end{array}$$

In equations (1) and (2), *λ* is the probability of information transmission, and *S*(*t*) and *I*(*t*) represent the proportions of susceptible and infected persons at time *t*. The SIS model includes the infected and the susceptible population, but their transmission modes are different. In the SIS model, the transmission is performed from the infected to the susceptible. There is also a situation where the infected are cured of the susceptible [29]. The calculation equations of the SIS model are as follows:

(3) $$\begin{array}{c} \frac{dS\left(t\right)}{dt}=\beta I\left(t\right)-\lambda S\left(t\right)I\left(t\right), \end{array}$$

(4) $$\begin{array}{c} \frac{dI\left(t\right)}{dt}=\lambda S\left(t\right)I\left(t\right)-\beta I\left(t\right). \end{array}$$

In equations (3) and (4), *β* is the probability of the infected becoming susceptible. The SIR model includes the infected, susceptible, and immune populations. It shows the process from the susceptible to the infection to the immune, which will no longer be infected [30]. The calculation equations are as follows:

(5) $$\begin{array}{c} \frac{dS\left(t\right)}{dt}=-\lambda S\left(t\right)I\left(t\right), \end{array}$$

(6) $$\begin{array}{c} \frac{dI\left(t\right)}{dt}=\lambda S\left(t\right)I\left(t\right)-\mu I\left(t\right), \end{array}$$

(7) $$\begin{array}{c} \frac{dR\left(t\right)}{dt}=\mu I\left(t\right). \end{array}$$

In equations (5)–(7), *μ* is the probability that the infected person will become immune.  Figure 5 shows the SI model, SIS model, and SIR model principles.

The article "Information Dissemination Model in Rural Live Broadcasting under Blockchain in the Era of Artificial Intelligence" was retracted in 2023. Reasons: unreliable results or conclusions; concerns about the data; concerns about the peer review; concerns about the citations.

SI, SIS, and SIR models described in Figure 5 are mainly used to represent the infectious disease information dissemination model. In addition to the infectious disease model, the information dissemination model also includes the influence model and the game-based information dissemination model. The former mainly refers to the impact on information dissemination, and the latter mainly refers to the specific relationship between information producers and disseminators. The SI model is suitable for diseases involving only susceptible and infected people and will not occur repeatedly. The susceptible person is infected immediately after effective contact with the infected person, without an incubation period, cure, and immunity. By comparison, the SIS model is a transmission model, an abstract description of the transmission process. It is applied to infectious disease transmission and information transmission research fields. The SIS model of infectious diseases assumes that the infected individuals at the source of infection (recorded as infected or I) pass the infectious diseases to the susceptible individuals (recorded as susceptible or S) through a certain probability. The infected individuals return to the susceptible state with a certain probability. On the other hand, once the susceptible population is infected, they will become a new source of infection and start circulating transmission. Lastly, SIR applies to susceptible, infected, and rehabilitated people. Rehabilitated people have only temporary immunity. They become susceptible after unit time and may be infected again [31]. Therefore, describing the current form of network information dissemination through the above model is very reasonable.

## 4. Information Dissemination Model under BT

The information dissemination model implemented under BT can help establish a more secure, reliable, and orderly storage technology for information dissemination. Users can review their communication information and its preciseness in information dissemination on the social network platform. Because BT's social network platform mechanism is reliable, it has become promptly popular [32]. The BT model has more user management, information dissemination, and system management advantages than traditional social networks. First, BT can control public discourses in the information dissemination between user nodes. Second, the protection measures for users are perfect, and they provide users with a safe and reliable information dissemination platform. In addition, the BT model also has a reward and punishment system for information transmission and implements reward and punishment measures for users who spread information according to the rewards and punishment. Finally, the information dissemination platform based on BT has a reputation system to judge the reputation of users in information dissemination and determine whether to implement specific control measures through the judgment results [33]. Based on the above, it is concluded that BT can provide technical support for the network information dissemination platform and promote the positive development of the rural live broadcasting system.  Figure 6 shows the principle and characteristics of BT's network information dissemination platform.

As shown in Figure 6, the transmission between BC user nodes is guaranteed by security measures for information transmission activities. Therefore, this work establishes a network information dissemination model through the BC. When the model is used for information dissemination, it is evaluated by the infectious disease model. The users include infected, susceptible, latent, and immune people, simulated through the susceptible exposed infected recovered (SEIR) model. The SEIR model adds latent individuals to the SIR model. It applies to diseases with latent period and lifelong immunity after curing in four groups: susceptible, exposed, infected, and rehabilitated. The susceptible person becomes the exposed person after effective contact with the infected person. The exposed person becomes the infected person after the average incubation period. The infected person can be cured and become a rehabilitated person. The rehabilitated person is no longer susceptible for life.  Figure 7 shows the main dissemination modes of the BC-optimized SEIR model.

The article "Information Dissemination Model in Rural Live Broadcasting under Blockchain in the Era of Artificial Intelligence" was retracted in 2023. Reasons: unreliable results or conclusions; concerns about the data; concerns about the peer review; concerns about the citations.

Figure 7 shows that the SEIR model is relatively perfect than other infectious disease models, making the information dissemination process more reliable. Moreover, different information disseminators can be transformed, and the calculation equations are as follows:

(8) $$\begin{array}{c} \frac{dS\left(t\right)}{dt}=-\lambda S\left(t\right)I\left(t\right), \end{array}$$

(9) $$\begin{array}{c} \frac{dE\left(t\right)}{dt}=\lambda S\left(t\right)I\left(t\right)-\delta E\left(t\right), \end{array}$$

(10) $$\begin{array}{c} \frac{dI\left(t\right)}{dt}=\delta E\left(t\right)-\mu I\left(t\right), \end{array}$$

(11) $$\begin{array}{c} \frac{dR\left(t\right)}{dt}=\mu I\left(t\right). \end{array}$$

In equations (8)–(11), *λ* is the probability of changing from the susceptible to the exposed. *δ* is the probability of changing from the exposed subject to the infected. *μ* is the state from the infected to the immune. This model evaluates the implemented BT model, and its development process of rural live broadcasting under BT is verified.

## 5. Evaluation of Information Dissemination Model in Rural Live Broadcasting

### 5.1. Evaluation of the Traditional Information Dissemination Model

With the development of rural networks, live broadcasting has been popularized in rural areas. Selling rural characteristic agricultural products is the main task in rural living broadcasting. However, in information transmission, their responses are different from those in urban areas when they promote their products in live broadcasting. Sometimes, what they do or say violates the current social values, which greatly impacts information dissemination. The infectious disease model describes the traditional rural live broadcasting.  Figure 8 shows the data of the traditional information dissemination model.

Figure 8 shows that the number of infected people in the SI model is almost zero at the initial information dissemination stage, and the susceptible proportion is almost 1. When the infection begins, the proportion of the infected increases, but the number of the susceptible is gradually decreasing. In about 20 days, almost all the susceptible are infected. In the SIS model, the initial states are similar to the SI model. The number of the infected almost reaches the upper limit in about 20 days. However, the number of the infected is not close to zero, indicating that someone will change from infected to susceptible. In the SIR model, there is an immune population. Almost everyone becomes immune when the infection lasts about 40 days, while the number of infected and susceptible is nearly zero.

The article "Information Dissemination Model in Rural Live Broadcasting under Blockchain in the Era of Artificial Intelligence" was retracted in 2023. Reasons: unreliable results or conclusions; concerns about the data; concerns about the peer review; concerns about the citations.

## 6. The SEIR Model under BT

The impact of information dissemination can be indirect. That is, it cannot intuitively describe the harm of information dissemination to the population. Therefore, it is necessary to comprehensively evaluate the impact of information dissemination on the population through factor analysis. The analysis of the effects of the SEIR model on information dissemination is more comprehensive than other models. Its specific impact on the information dissemination of the SEIR model needs to be considered under BT.  Figure 9 shows the comparison between the data evaluation of the SEIR model under BT and the traditional SEIR model.

As shown in Figure 9, BT has no impact on the transmission data of the SEIR model. The traditional SEIR model and the BT-optimized SEIR model analyze the information transmission data through infected, latent, susceptible, and immune people. The data display mode is the same, similar to the SIR model. Meanwhile, almost all people infected by information dissemination have become immune under both the traditional SEIR model and the BT-optimized SEIR model. Remarkably, the turning point of latent, susceptible, and immune people is about 20 days. In 20 days, the number of susceptible people is gradually cleared. The number of latent people peaks and then drops rapidly. The number of cured people also begins to rise rapidly. However, the number of infected people has increased accordingly, and the turning point appeared in about 30 days. The number of the infected begins to decline. Therefore, adding BT will not impact the overall dissemination scale of the SEIR information dissemination model. The proposed BT-optimized SEIR model aims to control the impact of information dissemination and control the impact of rumor dissemination on people. Thus, the impact of BT on information dissemination control needs to be considered.  Figure 10 shows the specific control status of the BC-optimized information dissemination model.

The article "Information Dissemination Model in Rural Live Broadcasting under Blockchain in the Era of Artificial Intelligence" was retracted in 2023. Reasons: unreliable results or conclusions; concerns about the data; concerns about the peer review; concerns about the citations.

In Figure 10, the SEIR model is the traditional SEIR model. The ASEIR model is the model with the reward and punishment system added to the traditional SEIR model. The BSEIR model is the SEIR model under BT. Through data analysis, it is found that after the reward and punishment system is added to the SEIR model, the maximum proportion of the model to false information is reduced by about 9% compared with the maximum value of the traditional SEIR model, and the duration is reduced by about ten days. In the forward information dissemination, the BSEIR model increases by about 10% more than the traditional SEIR model, and the duration increases by about 15 days. Compared with the traditional SEIR model, the proposed BT-optimized SEIR model reduces the maximum proportion of false information by about 13% and the duration by about 15 days. Compared with the traditional model, the maximum proportion of the positive information in the proposed BT-optimized SEIR model increases by about 19%, and its duration increases by about 30 days.

## 7. Conclusion

With the continuous promotion of the digital economy in recent years, AI has developed rapidly and is deeply integrated with various application scenarios. AI has gradually become an important technology to promote the development of economic innovation. In order to use AI to promote rural economic development and ensure the stable development of rural areas, this work discusses the information dissemination mode of rural live broadcasting under BT. The results are as follows: first, among the infectious disease models selected in this work, the proposed BT-optimized SEIR model can evaluate the overall impact of information dissemination on the population more accurately than SI, SIS, and SIR models. Therefore, this work designs the BT-optimized SEIR model to reflect the basic form of information dissemination through different types of people. Second, the proposed BT-optimized SEIR model does not affect the propagation process of the traditional SEIR model. BT optimization will not affect SEIR model basic information dissemination factors and dissemination process. Finally, an experiment is designed to compare the transmission data between the BT-optimized SEIR model, the SEIR model with a reward and punishment system, and the traditional SEIR model. As a result, the proposed BT-optimized SEIR model is much better than the other two information transmission models in controlling false information, positive information transmission efficiency, and duration. Therefore, using BT to optimize the information dissemination model does not affect the fundamental factors of information dissemination and controls the dissemination efficiency and duration of false information and positive information through its reward and punishment system and reputation system. The proposed BT-optimized SEIR model can comprehensively rectify the deterioration of information dissemination in rural live broadcasting. Additionally, this work helps create a more positive atmosphere for live information dissemination in rural areas. Compared with traditional information dissemination technology, the BT-optimized SEIR model has strong advantages in information dissemination speed. It safeguards information dissemination and comprehensively improves the current situation of network information dissemination. Finally, the research limitation is that too few factors are involved in the overall model evaluation. Future work will increase the research on the information dissemination model under more evaluation factors.

The article "Information Dissemination Model in Rural Live Broadcasting under Blockchain in the Era of Artificial Intelligence" was retracted in 2023. Reasons: unreliable results or conclusions; concerns about the data; concerns about the peer review; concerns about the citations.

## Figures and Tables

**Figure 1:** Principle of network platforms. (a) Stands for the audience; (b) for an anchor; (c) for the platform.

**Figure 2:** Selling mode of characteristic rural products in rural areas. (a) Selling the product by peasants themselves; (b) selling the product by public welfare anchors or other anchors.

**Figure 3:** Ways and main functions of rural live broadcastings.

**Figure 4:** Structure of a BC. (a) The overall principle; (b) the individual principle.

**Figure 5:** Three models of infectious diseases. (a) SI model; (b) SIS model; (c) SIR model.

**Figure 6:** Social networking platform under BT.

**Figure 7:** Basic principle of the SEIR model.

**Figure 8:** Information dissemination of the infectious disease model. (a) SI model; (b) SIS model; (c) SIR model.

**Figure 9:** Evaluation and comparison of the data in the SEIR model. (a) The traditional SEIR model; (b) the SEIR model under BT.

**Figure 10:** Evaluation of the dissemination data of the SEIR model under different conditions. (a) False information dissemination; (b) positive information dissemination.

## Data Availability

The data used to support the findings of this study are included within the article.
